The article "Comparative Numerical Analysis between Two Types of Orthodontic Wire for the Lingual Technique, Using the Finite Element Method" was published in 2021. Journal: Appl Bionics Biomech.

# Comparative Numerical Analysis between Two Types of Orthodontic Wire for the Lingual Technique, Using the Finite Element Method

**DOI:** 10.1155/2021/6658039

**Published:** 2021-03-25

**Authors:** Rosa Alicia Hernández-Vázquez, Rodrigo Arturo Marquet-Rivera, Octavio Alejandro Mastache-Miranda, Angel Javier Vázquez-López, Salvador Cruz-López, Juan Alejandro Vázquez-Feijoo

**Affiliations:** ^1^Universidad Politécnica del Valle de México, Departamento de Mecatrónica, Av. Mexiquense s/n Esquina Av. Universidad Politécnica, Col. Villa Esmeralda, Tultitlán, C.P. 54910 Estado de México, Mexico; ^2^Instituto Politécnico Nacional, Escuela Superior de Ingeniería Mecánica y Eléctrica, Sección de Estudios de Posgrado e Investigación, Unidad Profesional Adolfo López Mateos “Zacatenco”, Avenida Instituto Politécnico Nacional s/n, Edificio 5, 2do. Piso, Col. Lindavista, C.P. 07320 Ciudad de México, Mexico

## Abstract

In the lingual orthodontic technique, there are two paradigms regarding the type of wire used. Regardless of the material or gauge, some orthodontists choose to use the straight wire and resin and bond it to the surface of the tooth; they call it compensations. Other orthodontists prefer to bend the wire, giving it a mushroom shape. There is no specific indication for the use of each type of wire, so orthodontists use them according to their criteria. The present study establishes the bases so that it is possible to find the indications for each type of wire. A clinical trial of a lingual orthodontic patient was used. To carry out the comparative study, a straight arch was placed in his right arch and a mushroom arch in the left arch. Using 3D imaging, a high-biofidelity biomodel of the patient's mandible was generated, with which the FEM analysis was performed, which allowed comparing the reactions of the mandibular bone and appliances with the different arches. It was found that, on the side with the straight arch, there were greater deformations, and in the mushroom arch, there were greater stresses. With this, it is possible to find which clinical cases in each type of wire are indicated.

## 1. Introduction

Orthodontic treatments are generally requested by patients, for aesthetic reasons, considering that the smile and front teeth are socially associated as a fundamental part of a person's appearance, development, and social status. The importance of its correct occlusion in its physiological function is the least considered. These are reasons why parents worry about their children getting this benefit, so not long ago orthodontics was considered an exclusive treatment for children and teenagers. In countries like Mexico in many cases, these treatments are well accepted mainly by teenagers, who, despite the visibility of the brackets, consider it a sign of high social level [1].

That is why orthodontic treatment is helpful to achieve that aesthetic that is believed necessary for life in society. But this is only one of its benefits; although it is true that aesthetics are fundamental in social demands, orthodontic treatment fulfills an important function, in which it returns and improves a better functioning of the stomatognathic system. Mainly, the orthodontic treatment is aimed at bringing the teeth to their ideal position (or as close as possible) by remodeling the alveolar bone and thus improving facial aesthetics, and it also allows increasing the physiological life of the teeth, since it locates them in a position of equilibrium with respect to the surrounding forces and receiving the forces of mastication in the vertical and axial directions [2].

In addition, orthodontics establishes interactions with other areas of dentistry that allow better treatments. An example of this interaction is the one that is established between the prosthesis and oral rehabilitation when the replacement of teeth is necessary. Orthodontic treatment can be indicated to give the best conditions to the prosthesis (abutment parallelism, occlusion balance, anterior guide, canine guide, etc.) (Figure 1). This in turn improves the chewing, digestive, nutritional, and respiratory function, as well as the patient's affective, psychological, and emotional aspects [3].

As already mentioned, today, orthodontic treatment in adults is common. However, they tend to have greater resistance to treatment. They have lower tolerance to pain, and they demand to know more about the interventions they should undergo, time, cost, duration and frequency of appointments, and how to evaluate the effectiveness of the treatment, in other words, the results [4]. But mainly, unlike teenagers, they do not like to wear visible brackets, whether metallic or aesthetic. For this reason, invisible aesthetic orthodontics meets the expectations of this type of patient. The technique with lingual appliances has been in development for approximately 25 years, and with the experience of the cases treated, a completely protocolized technique has been conceived [5] (Figure 2).

Orthodontic tooth movement is a physical phenomenon in which the mechanical forces applied to the tooth are translated into biological events that occur in the cells and the extracellular matrix that surrounds them. The experimental orthodontic movements in rats induce dynamic changes in the nerve fibers and the density of the pulp blood vessels, which correspond to the sequence of changes observed in both the periodontal ligament and the alveolar bone [6]. These forces are generated by the bracket and directed through the wires or arches. In the case of the lingual technique, there are two types of arches that are commonly used: the straight and mushroom-shaped arcs. On this aspect, it is worth mentioning that there is still no accepted consensus or well-founded research, which has allowed establishing the criteria that allow selecting the one indicated for each specific case (Figure 3). There is a publication that mentions that orthodontists consider that the mushroom-shaped arch serves to compensate for the morphology of the lingual faces of the teeth when there is dental crowding. However, this leads to complicated biomechanics in some cases, as it requires precise bending, which often results in discomfort for the patient. In addition, they require many bends, which depend on the ability of the orthodontist to shape them precisely, which entails more work for him and time to prepare. With the straight arch, orthodontists believe that not only is it easier and faster to work with this arch but also the mushroom-shaped system presents some difficulties in its construction [7]. So, orthodontists use them, according to their criteria.

Knowing the magnitudes of the appropriate forces for each case is of utmost importance to minimize undesirable reactions both in the dental organ and in its tissues that make it up and other surrounding tissues [8]. One way to obtain the calculation and the reactions of the forces that occur is through analysis using the finite element method (FEM). This numerical method simulates a real physical phenomenon, through a geometric model, discretizing or dividing it into small parts called finite elements. These allow modeling structures with complex geometries which are divided into these small parts, in the form of triangles, squares, or tetrahedral whose vertices are joined to form nodes (Figure 4). In each of these nodes, the solution to the study variables is located through the equations that govern the phenomenon analyzed (elasticity, stresses, deformations, and elongations, among others). The number of finite elements that structure the geometry determines the precision of the analysis and simulation of reality and therefore the results [9].

A fundamental part for carrying out this type of simulation and analysis is the geometric model that is used. In the case of biological structures, these models that will represent the tissue or organ are called biomodel, which is the virtual three-dimensional representation of the biological structure [10–12]. The quality of this biomodel turns out to be fundamental for the analysis by FEM, since the biofidelity that it has [13–15] will allow the generation of the quantity and quality of the appropriate finite elements.

Initially, the biomodels were no more than representations of the structures through geometric figures that were far from representing their morphology and morphometry. Currently, 3D imagenology (magnetic resonance, standard computed tomography, and cone-beam tomography) is possible to generate these biomodels with high biofidelity, through various CAM/CAD-type computational systems (Figure 5) [16].

Simulation and analysis consist of the study of the biomodel that represents the biological element, in real situations in terms of its function and the agents that act on them. This simulation refers to the fact that, in the computer program, the biomodel is capable of reproducing or emulating the function performed by the biological structure. In addition, the biomodel can also simulate the biological response to agents outside it (pathologies, prostheses, forces, devices, etc.).

In the medical and dental area, the use of the FEM is relatively new; it is not quite common for the generality of doctors and dentists to handle this type of research methodology. Its application is a good tool to be able to predict and calculate, among many other applications in the various areas of dentistry, the results of the orthodontic forces applied in a treatment and in this way provide patients with better treatment plans. In this way, it is possible to meet the expectations of patients, especially adults.

Specifically, in the lingual technique as already mentioned, there are two types of arches or wires that are used: mushroom-shaped or straight. The selection of the caliber depends on the stage of the treatment. However, the choice of the arch shape depends on the criteria of the orthodontist, since there is no specific indication for each arch shape, in relation to the type of patient or case.

The present work shows through the application of this method the analysis of the types of arches used for lingual orthodontics. The objective is to find a numerical support that serves as a basis to establish, in a more objective way, which cases in each of the different wires should be used, depending on the stresses and reactions in the bone, the dental organs, and the wire itself.

## 2. Materials and Methods

For the numerical analysis that was carried out in the present work, a clinical case belonging to the CONRICYT Torre Médica Metropolitana, in its Orthodontic Research Department under the DDS MS Alfredo Gilbert Reisman, was used. This is a 29-year-old male patient who required lingual orthodontic treatment. His Ricketts analysis shows that he has a severe dolico facial pattern with bone class II. The molar relationship shows class I dental and canine class II dental relationship. The upper molar position is in class III with labial protrusion. In the Roth-Jarabak analysis, mandibular retrognathism is indicated. The diagnosis is skeletal and dental class II with open bite (Figure 6).

For the generation of the high-biofidelity biomodel, which is necessary to perform the numerical analysis, three-dimensional imaging of the patient was used. From Cranial Digital Volumetric Tomography (DVT) with the Cone-Beam Computed Tomography (CBTC) system, DICOM images are obtained that allow 3D reconstruction. This system is used to obtain images in tissues that are difficult to visualize. It is widely used in medicine and dentistry in the craniofacial region. This new imaging modality offers accurate and high-quality three-dimensional representations of the elements present in the maxillofacial complex. Unlike conventional tomography that shows consecutive slices, the data obtained by a DVT and processed by the computer creates a reconstruction of the studied volume.

### 2.1. FEM Analysis Considerations

To carry out this study, the biomodel of the patient's mandible was generated from his cone-beam tomography (Figure 7). The biomodel generated is shaped up of five different materials: dental organ, cortical bone, bracket, steel wire (stainless steel), and resin or adhesive.

After obtaining the biomodel, it was corrected and solidified using CAM/CAD-type computer programs, to be subjected to analysis. Once this was done, the controlled discretization of the same was carried out (Figure 8), obtaining a total of 1377416 elements and 2178470 nodes. It has high-order tetrahedral elements (Table 1).

The characteristics of the biomodel are described in Table 1, and the mechanical properties of the tissues are described in Table 2.

To carry out the simulation, the tissues are considered materials that present a linear-elastic behavior and whose internal structure is isotropic and homogeneous. Regarding border conditions, these were established around the mandibular condyles. Therefore, the displacements and rotations in the directions of the *X*, *Y*, and *Z* axes were restricted, in the anatomical region corresponding to the mandibular condyles. The applied force corresponds to those established by Jarabak as optimal forces [26], being distributed as follows: incisors and canines, 0.2 N; premolars, 0.5 N; and molars, 1.2 N. The *ANSYS®* computer program was used to perform the numerical analysis (Figure 9).

## 3. Results

Once the simulation and the numerical analysis had been performed, the total deformations and the normal and von Mises stresses that occurred in the complete system (mandibular bone, dental organs, brackets, and wire), the mandibular bone, and the wire were obtained, with both types of arch (mushroom-shaped and straight), obtaining the following.

In the complete system (Figure 10), it is observed that the maximum deformations (0.011 mm) occur in the dental process, in the mandibular border zone. Mainly to the left side where the mushroom arch was placed, the minimum deformations equal to 0 mm are found, in both condyles from the neck to their upper edge.

In the deformations in the analyses that only consider the mandibular bone (Figure 11), the results and the reactions are practically the same as those obtained in the complete system.

Specifically, in the wire (Figure 12), it is shown that the maximum deformations (0.009 mm) occur in the anterior teeth area, mainly towards the right side where the arch is straight. Minimum deformations (0.007 mm) occur on both sides (straight and mushroom-shaped), in the molar area. This is similar to the results and reactions presented by the deformation in the complete system and in the mandibular bone; only the distribution shows slight variations.

In the results of normal stresses and their reactions, the following was obtained. The normal stresses on the *X* axis in the complete system (Figure 13) show that the maximum stresses (3.11 MPa) are presented on the left side, where the arc has a mushroom shape. These stresses are in tension and are located in the upper right angle of the central incisor bracket. The minimum stresses (-2.22 MPa) occur on the right side (straight arch) and are compressive stresses disposed at the junction of the wire with the canine bracket.

Figure 14 shows that the maximum stresses in the *Y* axis (-5.20 MPa) are presented on the left side, on the mushroom-shaped wire, specifically at the union of the canine bracket with the wire, which are in compression. The minimum stresses (3.73 MPa) that are in tension are located on the right side, where the arch is straight, at the junction of the wire with the canine bracket.

Figure 15 shows that the maximum and minimum stresses on the *Z* axis are located on the left side, where the arc is in the mushroom shape. Maximum stresses (-4.49 MPa) are present in compression at the union of the wire with the lateral incisor bracket. The minimum stresses (2.74 MPa) are tensile stresses and are settled at the junction of the wire with the central incisor bracket.

Figure 16 shows that the maximum stresses on the *X* axis in the mandibular bone (0.48 MPa) are in tension and appear on the left side (mushroom-shaped wire), in the furcation crotch area of the first molar. The minimum stresses (-0.30 MPa) are in compression and occur on the right side (straight arch), in the alveolar process of the first premolar in its proximal area.

Figure 17 shows the maximum stresses on the *Y* axis in the mandibular bone (-0.81 MPa). They are in compression and occur on the left side (mushroom-shaped wire), in the alveolar process of the first molar, in its distal area. The minimum stresses (0.78 MPa) are in tension, on the right side (straight arch), in the alveolar process of the first premolar, in its proximal area.

Figure 18 shows that the maximum stresses on the *Z* axis in the mandibular bone are in tension (1.05 MPa) and the minimum (-0.73 MPa) in compression. Both appear on the left side (mushroom-shaped wire), in the furcation crotch area of the first molar. The maximum stresses are towards the distal are and the minimum towards the proximal are.

Figure 19(a) shows the stresses on the *X* axis in the wire. The maximum stresses (1.93 MPa) which are in tension are located on the right side where the mushroom arch is located, between the canine and the 1st premolar. The minimum stresses (-1.75 MPa) are in compression, and they are located in the central zone.  Figure 19(b) shows the *Y* axis stresses in the wire. The maximum stresses (-0.46 MPa) are shown on the right side where the mushroom arch is located, between the canine and the 1st premolar, which are in compression. The minimum stresses (3.37 MPa) are in tension and are around the right side, where the arch is straight.  Figure 19(c) shows the normal stresses on the *Z* axis in the wire. The maximums stresses which are in compression (-3.09 MPa) are observed in the molar area on the right side, where the mushroom arch is located. The minimum stresses (3.73 MPa) are in tension and are around the right side.

Finally, Figure 20 shows von Mises stresses throughout the system. The maximum values (7.64 MPa) are found on the right side (straight arch), at the junction of the wire and the canine bracket. In Figure 21, the maximum von Mises stresses (1.34 MPa) in the mandibular bone are presented on the left side (mushroom-shaped wire), in the alveolar process of the first molar, in its distal area.  Figure 22 shows that the maximum von Mises stresses in the wire (6.77 MPa) occur in the area where the mushroom-shaped wire is located in the first premolar.

## 4. Discussion

In the present work, the results and reactions obtained in the displacements, normal stresses, and von Mises stresses that occur in what was named the complete system (bone mandibular, dental organs, brackets, and wire) were analyzed. These results were compared with those found in the mandibular bone separately and in the wire, which is mushroom-shaped on the left side and straight on the right side. This allowed finding the following.

The deformations were increased on the side where the straight wire is located, in the three entities analyzed (Figure 23).

Figure 24 shows the stresses generated on the *X* axis. On the contrary to the deformations, the stresses are greater on the side where the wire has a mushroom shape, this result being consistent in the three entities analyzed (the complete system, mandibular bone, and wire). The same happens in the forces that are generated on the *Y* axis and the *Z* axis (Figures 25 and 26).

In the case of von Mises stresses (Figure 27), like deformations, the highest values are presented on the side where the straight wire is located, this result being consistent in the three entities analyzed (the complete system, the mandibular bone, and the wire).

Both the deformations and the von Mises stresses are greater when using the straight arch. This is consistent since the von Mises criterion is the most conservative and is related to the strain energy. That is why it is logical that the results of these two analyses are congruent.

On the other hand, the stresses generated in the mushroom-shaped wire are greater than those of the straight wire, and these stresses are transmitted to the mandibular bone and the brackets and wires. The areas where the maximum stresses occur in the mushroom wire correspond to the places where the geometry of the mushroom is formed (where the bends of the wire are made for the conformation of the mushroom). By bending the wire so that it acquires this shape, stress concentrators are being generated, due to its geometry. This concentration is transmitted to the bone and other adjacent elements, a situation that does not occur in the straight wire. As there are no such stress concentrators, only deformations of the agents and loads to which the wire is subjected are presented, and therefore, the stresses generated and transmitted are lower.

According to this, it is possible to affirm that, when using a straight wire, less stresses will be generated that act on the bone and dental organs than if a mushroom-shaped wire is used. This is, at least, for this case study. Although this is a very subdued first approximation to reality, further studies of this type still need to be carried out. These studies should include a greater number of study subjects and make a greater limitation of the variables, which could be done by trying to ensure that the study subjects have similar characteristics (higher control of the inclusion and exclusion criteria) and that the study is carried out with complete arches. It is worth mentioning that this study is the first of others where the aspects are considered.

This is not to say that the present study does not establish a good starting point. On the contrary, this study establishes the bases where it is observed that biomechanically, there are differences between using a straight wire or a mushroom-shaped wire, as well as the possible repercussions that could be generated. As already mentioned, there is no documented support for the orthodontist to decide which is better or which cases in each one are indicated. With studies of this type, the consensus not yet reached can be achieved, with proven scientific bases, rather than through personal preferences or empirical knowledge. In addition, it demonstrates the usefulness of using the finite element method in dental research, as a tool that could reduce the time and number of study subjects.

## 5. Conclusions

Based on the previous discussions, it was possible to reach the following conclusions.

The straight wire transmits less stress than a mushroom-shaped wire, which would be important to consider since such stresses could lead to undesirable movements during treatment. Some of these efforts are located in anatomical areas of importance to consider during orthodontic treatment. These areas were stresses within the alveolus of the first molar, in the furcation area and in the alveolar ridge.

Considering that lingual orthodontics is mostly used by adults, the condition that these stresses exert on the alveolar and supporting bone is an important point to consider. Adult patients may represent some conditions or habits that compromise periodontal health: osteopenia, osteoporosis in the case of women or metabolic and systemic diseases, smoking, and poor brushing techniques due to lack of time, which can affect the supporting tissues.

On the other hand, although with the straight arch the stresses are much lower, the deformations are also aspects to consider. The deformation of the wire can cause them to deactivate, or their action is not adequate. Above all, when patients do not attend their check-up appointments with the necessary regularity, which is known, it can also generate undesirable movements that later have to be corrected when they go to their appointment and that delay the treatment time or have to consider other circumstances in addition to the initial treatment plan.

This is clear for orthodontists: greater stress on bone and anatomical areas and greater damage to supporting tissues; therefore, in patients with periodontal conditions, it can cause problems (this depends on age, sex, diet, dentition, health status, etc.). The mushroom arch causes greater stresses on bone and anatomical areas, which could contraindicate its use in this type of patient.

A deformation of the wires demonstrates that there is no control in the mechanobiology and mechanotransduction of orthodontic movement. For patients who do not come regularly, this can be a problem. The straight arch suffers from greater deformations, which would contraindicate its use in these cases.

## Figures and Tables

**Figure 1:** Contributions of orthodontics to better prosthetic treatments. Orthodontics verticalizes the position of the inclined teeth that will serve as pillars for the prosthesis, improving its support.

**Figure 2:** Standardized arches for the lingual technique: (a) mushroom shape and (b) straight. The choice of the type of arch is according to the criteria and experience of the orthodontist.

**Figure 3:** Mechanotransduction of the bone by the action of orthodontic forces. When the orthodontic forces produce the movement of the dental organ, on the side towards which these forces are directed, they cause the osteoclasts to activate, producing osteolysis of the bone. In the same way, on the opposite side, the osteoblasts are activated, producing bone osteogenesis.

**Figure 4:** Finite elements of low biofidelity models. The low biofidelity of the biomodels causes the results to be far from those obtained in reality.

**Figure 5:** First biomodels of dental organs.

**Figure 6:** Radiographic study (cranial lateral radiography and orthopantomography) and cephalometry (Ricketts analysis, Jarabak analysis, and soft profile analysis) of the patient, necessary for the diagnosis of the patient.

**Figure 7:** High-biofidelity biomodel of the patient, generated from the latest generation tomography, necessary to perform the numerical analysis.

**Figure 8:** Discretization of the patient's biomodel with brackets and wires in place, prior to performing the numerical analysis.

**Figure 9:** Boundary conditions and forces applied to the wire according to their actual application to brackets and teeth. The red arrows indicate the direction of the forces generated in the wire, in each dental organ.

**Figure 10:** Total deformation occurring in the complete system (mandibular bone, dental organs, brackets, and wires). The red marker indicates the maximum deformations, and the blue marker indicates the minor deformations.

**Figure 11:** Total deformation that occurs in the mandibular bone. The red marker indicates the maximum deformations, and the blue marker indicates the minor deformations.

**Figure 12:** Total deformation that occurs in the wire. The red marker indicates the maximum deformations, and the blue marker indicates the minor deformations.

**Figure 13:** Normal stresses in the *X* complete system (mandibular bone, dental organs, brackets, and wires). The red marker indicates the maximum stresses, and the blue marker indicates the minor stresses.

**Figure 14:** Normal stresses in the *Y* complete system (mandibular bone, dental organs, brackets, and wires). The red marker indicates the maximum stresses, and the blue marker indicates the minor stresses.

**Figure 15:** Normal stresses in the *Z* complete system (mandibular bone, dental organs, brackets, and wires). The red marker indicates the maximum stresses, and the blue marker indicates the minor stresses.

**Figure 16:** Normal stresses in *X*, mandibular bone. The red marker indicates the maximum stresses, and the blue marker indicates the minor stresses.

**Figure 17:** Normal stresses in *Y*, mandibular bone. The red marker indicates the maximum stresses, and the blue marker indicates the minor stresses.

**Figure 18:** Normal stresses in *Z*, mandibular bone. The red marker indicates the maximum stresses, and the blue marker indicates the minor stresses.

**Figure 19:** Normal stresses in the wire: (a) *X* axis; (b) *Y* axis; (c) *Z* axis. The red marker indicates the maximum stresses, and the blue marker indicates the minor stresses.

**Figure 20:** von Mises stresses on the complete system (mandibular bone, dental organs, brackets, and wires). The red marker indicates the maximum stresses, and the blue marker indicates the minor stresses.

**Figure 21:** von Mises stresses on the mandibular bone. The red marker indicates the maximum stresses, and the blue marker indicates the minor stresses.

**Figure 22:** von Mises stresses on the wire. The red marker indicates the maximum stresses, and the blue marker indicates the minor stresses.

**Figure 23:** Total deformations (mm). The graph shows a comparison between the deformations that were generated in each of the analyzed sections: complete system (mandibular bone, dental organs, brackets, and wires) and separately the mandible and the two different types of arches or wires.

**Figure 24:** Normal stresses in the *X* axis (MPa). The graph shows a comparison between the stresses in the *X* axis that were generated in each of the analyzed sections: complete system (mandibular bone, dental organs, brackets, and wires) and separately the mandible and the two different types of arches or wires.

**Figure 25:** Normal stresses in the *Y* axis (MPa). The graph shows a comparison between the stresses in the *Y* axis that were generated in each of the analyzed sections: complete system (mandibular bone, dental organs, brackets, and wires) and separately the mandible and the two different types of arches or wires.

**Figure 26:** Normal stresses in the *Z* axis (MPa). The graph shows a comparison between the stresses in the *Z* axis that were generated in each of the analyzed sections: complete system (mandibular bone, dental organs, brackets, and wires) and separately the mandible and the two different types of arches or wires.

**Figure 27:** von Mises stresses (MPa). The graph shows a comparison between von Mises stresses that were generated in each of the analyzed sections: complete system (mandibular bone, dental organs, brackets, and wires) and separately the mandible and the two different types of arches or wires.

**Table 1:** Characteristics of the biomodel.

Tissue	Biomodel
Mesh	Tetrahedral solid elements [12, 17–25]
Meshing	Semicontrolled
Mesh quality	High-order quadratic elements
Nodes	2178470
Elements	1377416

**Table 2:** Mechanical properties used in the analysis.

Tissue	Young's modulus (GPa)	Poisson's ratio
Enamel	70	0.30
Dentin	18.3	0.30
Cortical bone	15	0.32
Steel	193	0.29
Resin	12.4	0.30

## Data Availability

All data generated or analyzed during this study are included in this published article.
